# The Development of Illness Anxiety Disorder in a Patient After Partial Thyroidectomy

**DOI:** 10.7759/cureus.25416

**Published:** 2022-05-27

**Authors:** Neeraj Kancherla, Srija Chowdary Vanka, Sandesh Pokhrel, Reshma Bano Shahzadi, Ganipineni Vijaya Durga Pradeep

**Affiliations:** 1 Psychiatry, King George Hospital, Visakhapatnam, IND; 2 Psychiatry, Dr. Pinnamaneni Siddhartha Institute of Medical Sciences and Research Foundation, Chinna Avutapalle, IND; 3 Psychiatry, Nepal Medical College, Lalitpur, NPL; 4 Psychiatry, N.K.P. Salve Institute of Medical Sciences and Research Center, Nagpur, IND; 5 General Medicine, SRM Medical College Hospital & Research Center, Chennai, IND; 6 General Medicine, King George Hospital, Visakhapatnam, IND

**Keywords:** hypochondriasis, psychiatry, anxiety, somatoform disorder, illness anxiety disorder, mental health

## Abstract

The Diagnostic and Statistical Manual of Mental Disorders, Fifth Edition (DSM-5), characterises illness anxiety disorder (IAD) as the preoccupation with having or acquiring a serious illness in the absence of somatic symptoms (or, if present, symptoms that are only mild in severity). DSM-5 includes illness anxiety disorder in the category called somatic symptom and related disorders, characterised by prominent somatic concerns, distress, and impaired functioning. More often than in psychiatric settings, individuals with illness anxiety disorder are encountered in primary care and specialist medical settings. Despite negative laboratory results, the benign course of the alleged disease over time, and adequate reassurances from specialists, their conviction of being ill persists. Illness anxiety preoccupations are heterogeneous, and the degree of insight is variable. Their illness-related preoccupation interferes with their relationships with family, friends, and coworkers. They are frequently addicted to internet searches about their feared illness, inferring the worst from the information (or false information) they uncover. Patients with illness anxiety disorder often have comorbid psychopathology, especially anxiety and depressive disorders. Typically, illness anxiety disorder is chronic. Physical symptoms are absent or mild and frequently represent a misinterpretation of normal bodily sensations. This case report presents the case of a patient diagnosed with IAD by a psychiatrist. The patient had been seen by his primary care physician and therapist for three years without any improvement in his symptoms before he was referred to a psychiatrist. After undergoing a partial thyroidectomy in 2018, this patient has been experiencing increasing symptoms of recurrent anxiety/fear consistent with IAD, despite extensive medical examinations that have consistently revealed normal results.

## Introduction

Illness anxiety disorder (IAD; formerly known as hypochondriasis (HC), a term that has been renamed in the DSM-5 due to the detrimental connotation) is a psychiatric disease characterised by an overwhelming fear of having or developing a major undetected medical condition. The criteria for Illness anxiety disorder (IAD) are fulfilled by only about 26-36% of patients who have been diagnosed with hypochondriasis [1]. The patient's distress stems mostly from an unjustified fear of having a disease rather than physical symptoms, and it remains despite a negative physical examination and laboratory testing. Physical symptoms are absent or mild, and they frequently indicate a misinterpretation of normal bodily responses [2]. Due to its recent inclusion in the DSM-5, which was published in 2013, illness anxiety disorder's prevalence cannot be accurately estimated. Based on a meta-analysis of 12 studies, the prevalence of illness anxiety disorder among medical outpatients (e.g., family practice and primary care) is approximately 0.75% [1]. The exact etiology of IAD is mostly unknown. The cognitive-behavioural model has been experimentally well demonstrated among the different psychological theories that describe how patients develop illness anxiety, which leads to an effective approach to treatment [3]. According to this model, dysfunctional beliefs about bodily symptoms and illness play an important role in developing illness anxiety. A fear of illness dominates the opinion of practitioners regardless of a lack of symptoms or positive test findings. The purpose of a visit to the medical practitioner is to obtain confirmation that they do not have the feared illness or to be reassured that it does not exist. It is possible to gain a different perspective on the pathology of the worry depending on the individual patient. While some patients can recognize their worries are excessive but are unable to curb them, others cannot be dissuaded from their fears of being ill [4,5]. Patients with maladaptive behaviour may frequently check themselves for skin problems, hair loss, or fear physical disabilities and may be oblivious to their social and occupational obligations, as a result of excessive body-checking practices [1]. A majority of IAD patients can be classified as either care-seeking or care-avoidant in nature. While a patient of the care-seeking type often gets multiple medical evaluations and medications and switches health care providers, the care-avoiding type usually avoids seeking medical attention for fear of being diagnosed with a life-threatening illness (e.g. diabetes mellitus, HIV) [6]. Patients with IAD might well be preoccupied with a specific diagnosis (for example, cancer, diabetes, or HIV infection), a physiological function (e.g., bowel movements), natural variation in function (e.g., in heart rate or blood pressure), or a vague physical experience (e.g., "weary heart"). The patient's concern can span multiple organ systems, and the emphasis of their attention may alter over time. While some patients might see that their concerns about their sickness are unwarranted, others remain steadfast in their beliefs [7]. Before diagnosing illness anxiety disorders, doctors must rule out other medical problems, particularly early phases of endocrine, immunologic, neurologic, oncologic, and rheumatologic diseases [1,4]. The present report describes a case involving a patient who developed IAD after undergoing a partial thyroidectomy. The disease course of the patient has been marked by recurring visits to the physician and therapist over the course of three years without improvement in the patient's signs and symptoms.

## Case presentation

History of the presenting complaint

The patient was a 31-year-old male immigrant to the US from El Salvador whose primary care physician referred him to the psychiatry hospital for a mental health evaluation. Since undergoing a partial thyroidectomy in 2018, the patient reports that his anxiety and fear of acquiring various diseases have increased. For the previous three years, he had experienced recurrent episodes of anxiety and panic attacks, as well as moderate somatic symptoms. He reports that every slight physical symptom causes him to panic to the extent that he experiences panic attacks and worries that he has a terrible illness. In addition, he has trouble falling asleep, diffuse muscle aches throughout the body, intermittent abdominal discomfort, and physical weakness. He has visited his physician numerous times, but he recognizes that his fears are unfounded. Six years ago, the patient was diagnosed with generalised anxiety disorder, for which he has been prescribed hydroxyzine and alprazolam, twice daily. After using alprazolam for a month, the patient quit out of concern for addiction and has since used hydroxyzine infrequently. He continued to feel anxious and had some somatic symptoms. A review of all the systems was normal. The patient has no psychiatric history in the family. The patient denied any manic or psychotic symptoms. A suicidal or homicidal ideation was also denied by the patient. There was no history of substance abuse, smoking or drinking. The patient has comprehensive medical examinations from his primary care physician regularly, after which he feels fine for a few months, but his anxiety and fear of acquiring an illness resurface later. The patient's physician had referred him to a therapist two years prior. After five sessions with the therapist, the patient has not seen any alleviation in symptoms. Consequently, he discontinued therapy later. His symptoms had increased again in the month preceding the current presentation; therefore, he was referred to the psychiatrist.

Examination

A mental status assessment revealed a clean and well-groomed middle-aged man. His demeanour was cooperative, calm, and he made eye contact appropriately. He interacted rationally during the interview. There were no problems with his speech. His mood was described as anxious with congruent affect. He has a normal range and intensity, and he is not labile. He had a simple, linear thought process. Suicidal or homicidal thoughts were not present. There were no reports of delusions or hallucinations. His insight, judgement, memory, and concentration were all good. He was awake, alert, and aware of his surroundings, including time, location, people, and events. He has a normal gait and station.

## Discussion

Illness anxiety disorder is a diagnosis of exclusion. Ideally, a patient should undergo a thorough physical exam and relevant tests appropriately suited to their symptoms before being diagnosed with IAD [1]. Currently, it is unclear what causes IAD. A number of risk factors have been implicated in its development, including having a family history of health anxiety, experiencing serious medical illness or having parents/siblings with serious medical conditions, having an underlying anxiety disorder (e.g., generalised anxiety disorder), spending excessive time researching health-related topics, etc. [6]. Adolescents are frequently affected by IAD with no prevailing gender pattern, and its severity typically worsens with age. Also, unemployment and undereducation increase the risk [1,8]. An observational study (n = 24) revealed that people with high levels of health anxiety focused more on body symptom words (e.g., dizziness, headache, and nausea) than people with low levels of health anxiety and that this attentional bias toward body symptom words was associated with rostral anterior cingulate cortex hypoactivity. Studies of biological correlates have found that compared with healthy controls, patients with hypochondriasis have decreased levels of plasma neurotrophin-3 and platelet serotonin and smaller pituitary volumes [9,10]. Our patient has a known diagnosis of generalised anxiety disorder, and he is not compliant with his medication. With the backdrop of a prior anxiety diagnosis, it is possible that having undergone a partial thyroidectomy surgery triggered IAD in him and made his anxiety worse. Often, he complained of vague somatic symptoms such as headache, abdominal pain, nausea, and myalgia, and feared that these symptoms are signs of an underlying serious illness.

IAD poses a significant risk of functional impairment. Clinically significant illness anxiety is associated with more workdays missed, more functional impairment, and higher use of disability benefits than general and medical populations without illness anxiety [11-13]. Based upon studies of hypochondriasis and the symptom of health anxiety, it is thought that illness anxiety disorder is often chronic with fluctuating symptoms [14]. At baseline, patients who are in remission display lower disease conviction, fewer somatic symptoms, improved functioning, and fewer disability days. During the months following medical consultation, our patient had only mild anxiety, very little or no somatic symptoms and was able to attend work without illness anxiety thoughts lasting from weeks to months.

It is possible to suspect that a patient has an illness anxiety disorder in primary care or general medical settings if they have had considerable medical care but are still unsatisfied with it when multiple physicians are consulted for the same condition with negative diagnostic evaluations and when medical attention exacerbates rather than eases the patient's concern over their health status [2]. Our patient has experienced many instances of recurrent worry about being diagnosed with a major disease, despite negative test results and assurances from the physician. Even the therapy sessions haven't been able to ease his anxiety. A majority of people with IAD are found in primary care settings rather than mental health clinics, leading to a delayed inception of treatment and, ultimately, a deterioration of their mental condition. Primary care physicians (PCPs) are often not trained to recognize the absence of physical symptoms in patients with IAD. Additionally, this wastes the physician's time and depletes scarce medical resources.

Few neuroimaging studies have examined the functional characteristics of patients with HC/IAD. Studies on activities involving executive function found that dorsolateral prefrontal cortex, striatum, and left thalamus were less active during executive function activities, while the amygdala was more active, suggesting hypoactivity of areas related to planning and executive function and increased activity of anticipatory fear regions. Compared to those who suffered from obsessive compulsive disorder (OCD) and panic disorder, these findings had no significant difference [15].

One of the most crucial aspects of treating IAD is building long-term trust between the doctor and the person they are treating [16]. It is important to recognize the worries and concerns that patients have. When it comes to the proper management of IAD, patient education is the most critical component. Providing patients with reassurance and information about typical physiological functions is a difficult balancing act that must be done carefully [17]. In order to prevent the overuse of the medical system, it is advisable to avoid performing additional imaging studies and seeking expert referrals after a serious medical illness has been ruled out. Primary care physicians should refer patients to specialist clinics in a compassionate, non-judgmental manner so that patients do not feel dismissed or abandoned. A regular schedule of follow-ups will reduce the number of trips to the emergency department and other medical providers. Psychotherapy is the first-line treatment for IAD [1]. Using cognitive-behavioural therapy (CBT) for health anxiety, patients learn to recognize and change unhealthy patterns of thinking and behaviour, as well as develop new explanations for their symptoms [18]. Three recent meta-analyses have found that CBT is an effective treatment for patients with high levels of health anxiety [17]. Recent "third-wave" CBT techniques for health anxiety include group acceptance and commitment therapy and individual mindfulness-based cognitive therapy [19,20]. There is minimal but promising evidence that psychopharmacologic therapies for health anxiety are beneficial. In a long-term follow-up assessment of hypochondriac patients treated with selective serotonin reuptake inhibitors, 60% of patients no longer satisfied HC criteria 8.6 years after the study ended [17]. The response rates for both fluoxetine and CBT in a large, randomised study involving 195 patients were 44.4% and 39.6%, respectively, with no statistically significant difference between the two treatments. The combination of the two medicines performed much better (47.2% response) [17].

Early referral for psychiatric evaluation is associated with a better prognosis for individuals with illness anxiety disorder than is general medical care alone. Our patient was managed by his PCP for three years without an appropriate diagnosis or referral to a psychiatrist, resulting in continuity of symptoms. Research has also shown that patients who are cooperative, tolerant, and optimistic have better outcomes. It may be possible to have a fair to favourable prognosis for IAD if the patient responds well to psychotherapy, medicine, or both. However, the prognosis becomes bleak if the patient has significant IAD symptoms and is resistant to psychiatric drugs and psychotherapy [11]. During the course of our patient's treatment, he is scheduled to undergo weekly CBT sessions as well as monthly outpatient visits to the psychiatrist and primary care physician. So far, his response to CBT has been positive as he has been cooperative and optimistic, and his anxiety symptoms have returned to baseline.

## Conclusions

In summary, we have a 31-year-old male with a history of generalized anxiety disorder who began experiencing recurrent symptoms of anxiety and fear. These symptoms have no identifiable medical etiology. Symptoms appear to have been triggered after partial thryoidectomy in the backdrop of known GAD. Given the non-specific nature of the symptoms, a delayed referral for psychiatric evaluation has caused the diagnosis to be delayed. It is critical for general physicians and family care physicians to understand illness anxiety disorder to be identified and treated effectively. General practitioners need to maintain IAD as a differential diagnosis. An assessment of the potential for the development of IAD following a major medical diagnosis or among patients with coexisting anxiety disorders must be made. 

It is essential to emphasise empathy, open dialogue, coordinated testing, and consistent delivery of information between the patient, the mental health practitioner, and the medical practitioner in order to prevent iatrogenic harm, unnecessary testing, and inappropriate treatment. As part of his treatment plan, our patient will undergo weekly CBT sessions as well as regular monthly visits to both his psychiatrist and primary healthcare provider.
